# Circ 003390/Eukaryotic translation initiation factor 4A3 promoted cell migration and proliferation in endometrial cancer via vascular endothelial growth factor signaling by miR-195-5p

**DOI:** 10.1080/21655979.2022.2069358

**Published:** 2022-05-12

**Authors:** Jing Ma, Xiwa Zhao, Li Shi

**Affiliations:** Department of Gynecology and Obstetrics, The Forth Hospital of Hebei Medical University, Shijiazhuang, China

**Keywords:** circWEE1, Endometrial cancer, miR-195-5p, EIF4A3, VEGF

## Abstract

The differential expression of circRNA in different biological samples renders it as an ideal biomarker for disease diagnosis and identification of tissue development. In addition, the gradual clarification of the mode of action of circRNA in disease makes it as a potential therapeutic target. The purpose of this study is to investigate the role and regulating mechanism of circular RNA has circ 003390 (circWEE1) on Endometrial cancer (EC) genesis. To estimate clinical values of circWEE1 on cell migration and proliferation in EC, and its possible mechanisms. The expression of circWEE1 and EIF4A3in EC cells have been evaluated using qPCR and Western blot. The expression of circWEE1 and EIF4A3 levels were increased in patients with EC. Over-expression of circWEE1 or down-regulation of miR-195-5p promoted cell migration and proliferation in EC. Next, we verified that eIF4A3 binds to the circWEE1 mRNA transcript, circWEE1 served as a sponge that directly targeted miR-195-5p. Bioinformatics prediction forecast that miR-195-5p directly targeted VEGF at 3’-UTR, which was confirmed by luciferase reporter assay. Our findings indicate that Circular RNA hsa circWEE1/EIF4A3 promoted cell migration and proliferation in EC via VEGF signaling by miR-195-5p, which could provide pivotal potential therapeutic targets for the treatment of EC.

## Highlights

- We identified that circWEE1 acts as an oncogene and promotes EC cell proliferation and migration.We identified that circWEE1 acts as an oncogene and promotes EC cell proliferation and migration.
- We found that CircWEE1 can directly bind to miR-195-5p and regulate its expression.
- We demonstrated that VEGF is target genes of the circWEE1/ miR-195-5p axis in EC cell.
- We provide pivotal potential therapeutic targets for the treatment of Endometrial cancer.

## 1. Introduction

Endometrial cancer (EC), one of the most common primary woman tumors, harbors extremely high morbidity and mortality [1]. Most EC patients were with early stage had good prognoses after the surgery, with only rare cases (10 ~ 20%) with poor prognoses [2]. At present, surgical resection is the preferred therapy of EC [3]. However, due to the highly invasion, rapid growth of EC, and easy-to-relapse, it is difficult to completely resect the tumor by surgery alone [3]. Clinically, surgery is often combined with radiotherapy, chemotherapy, interventional therapy, etc., however, the efficacy is still minimal [4]. Therefore, in-depth study of the pathological mechanism of EC from a molecular perspective is a hot topic and direction in this field, which provides clinical diagnostic markers and specific therapeutic targets of EC [4].

Vascular endothelial growth factor (VEGF), specific mitogen isolated from endothelial cells in the late 20th century, has been confirmed to have the ability of inducing both physiological and pathological angiogenesis [5]. In the past period, vascular permeability factor has become the most newly-discovered factor that promotes vascular permeability [6]. However, it has been later proved to be identical to VEGF after isolation and extraction [6]. VEGF is one of the most important pro-angiogenic factors, and VEGF/VEGFR signaling pathway plays a critical role in the pathological process of blood vessel growth [7]. Relevant studies have shown that oncogene transfection significantly increases angiogenesis activity by enhancing tumor VEGF expression [6,7].

Eukaryotic translation initiation factor 4A (eIF4A) protein, belonging to the DEAD-box RNA helicase family, has RNA-dependent ATPase activity and ATP-dependent RNA helicase activity [8]. Three types of eIF4A have been identified in vertebrates: eIF4A1, eIF4A2, and eIF4A3. Apart from participation in translation initiation, eIF4A family members also play an important role in multiple life processes, such as embryonic development. Although three types of eIF4As are highly similar in sequence, their functions are not the same [9]. The uniqueness and diversity of eIF4A members are usually regulated by interacting proteins. The initiation of translation is often out of control in cancer cells [9]. In transformed cells and cancer cells, the expression levels of many translation initiation factors, including eIF4A3, are altered, indicating that eIF4A3 may be involved in carcinogenesis and tumor progression, which is a potential therapeutic target [10].

MicroRNAs (miRs) are a class of non-coding small RNA molecules with approximately 19–24 nucleotides in length [11]. In 1993, the first miR lin-4 was discovered in Caenorhabditis elegans [12]. Ever since then, a large number of studies have shown that miRs regulate important biological activities in cells and organisms, including cell proliferation, growth, apoptosis, differentiation, and metabolism [13]. Meanwhile, miRs have been found to play a role similar to oncogenes or tumor suppressor genes [11]. To be specific, some miRs are abnormally expressed in tumors, which are closely associated with the occurrence and development of tumors [14]. In recent years, more and more studies have been performed on EC-associated miRNAs [15]. Most of the studies focus on analyzing miR expression profiles in EC tissues, and based on this, some specific changes in miR targets and related functions are also explored to investigate the roles and mechanisms of miRs in EC [16].

Circular Rs (circRs) are a class of circular non-coding RNAs generated by alternative splicing of precursor RNA, typically consisting of more than one exon [17]. CircR was first discovered in Sendai virus in 1976, then detected in yeast mitochondria and was first observed in human cells in 1993 [18]. For a long time since then, research on circR has been based on RNA viruses, while little attention has been paid to the research in eukaryotic cells [18]. With the development of transcriptomic gene sequencing technology, recent studies have shown the existence of circRs in animal cells, plant cell protozoa [17]. CircRs might be likely be a new generation of biomarkers or therapeutic targets, including in human disease diagnosis, treatment, and identification of tissue development [17]. Circ 003390 (circWEE1) was significantly up-regulated in gliomas and its level was positively correlated with high metastasis rate and poor prognosis in glioma patients [19]. CircWEE1 may play a carcinogenic role in the progression cancer. The knockout of circWEE1 reduced the viability, migration ability of tumor cells. The study estimated clinical values of circ 003390 (circWEE1) on cell migration and proliferation in EC, and its possible mechanisms.

The purpose of this study is to investigate the role and regulating mechanism of circular RNA has circ 003390 (circWEE1) on Endometrial cancer (EC) genesis and to estimate clinical values of circWEE1 on cell migration and proliferation in EC, and its possible mechanisms.

## 2. Materials and methods

### 2.1 Clinical tissue specimens

This study was approved by the Ethics Committee of the Forth hospital of Hebei Medical University (No. 2020KY065). All the serum samples were immediately snap frozen in liquid nitrogen and stored at −80°C for further using. Neuropathological evaluation was performed according to the WHO classification by two experienced clinical pathologists. Basic knowledge of patient with EC was showed at Table 1. All methods were carried out in accordance with relevant guidelines and regulations. Informed consent was obtained from all participants.

**Table 1.** Patients demographic data and characteristics

Variables	All patients (24)	All patients (24)
Age (yr)		
≤55	12	12
>55	12	12
Tumor size (cm)		
≤3.0	6	
>3.0	18	
Edmondson grade		
I–II	6	
III–IV	18	

### 2.2 RNA extraction and real-time PCR and microarray data

Total RNA was extracted using TRI-zol reagent (Invitrogen; Thermo Fisher Scientific, Inc.). cDNA was synthesized using a High-Capacity cDNA Reverse Transcription kit (Applied Biosystems, Foster City, CA, USA). qRT-PCR was performed using a SYBR Green kit (Bio-Rad Laboratories, Inc., Hercules, CA, USA) in an ABI 7900 PCR Thermal Cycler. The total volume of the amplification reaction system was 20 µl, including 6 µl primers, 10 µl of SYBR Green PCR Master Mix, 1.5 µl cDNA, and 2.5 µl ddH_2_O. PCR started at 95°C for 15 min, followed by 40 cycles at 95°C for 10s, 60°C for 40s, and finished by 40s at 60°C in the last cycle.

The primers used were

circWEE1: Forward (5´-GGATAAACCGTGGTAATTCTATG-3´) and Reverse (5´-GGCAAATGCTTTCGCAGTAG-3´);

EIF4A3: Forward (5´-AAGGGAGAGATGTCATCGCAC-3´) and Reverse (5´-GCTTGAGTTTCACGAACCTGA-3´);

GAPDH: Forward (5´-ATCTTCCAGGAGCGAGATCCC-3´) and Reverse 5´-TGAGTCCTTCCACGATACCAA-3´).

The mRNA expression levels of genes were measured using the 2ΔΔ-Ct method. GAPDH was used as internal control. Microarrays (HLivH180Su14) were purchased from Shanghai Outdo Biotech Co. Ltd. (Shanghai, China).

### 2.3 Cell lines and culture and cell transient transfection

The human EC cell lines (HEC-1-A, HEC-1B, KLE, Ishikawa) and normal human endometrial epithelial cells (hEM15A) were purchased from the Cell Bank of the Chinese Academy of Sciences. All cell lines were cultured in Dulbecco’s modified Eagle’s medium (DMEM; Life Technologies Corporation, Carlsbad, CA) containing 10% fetal bovine serum (FBS, Gibco) at 37°C, 5% CO 2, and 95% air. All oligonucleotides sequences were synthesized by Gene-Pharma (Shanghai, China). KLE or HEC-1B cells were transfected using the Lipofectamine 2000 Kit (Invitrogen, Carlsbad).

### 2.4 CCK-8 proliferation vitality assay

10 μL CCK-8 assay (Dojindo, Kumamoto, Japan) was carried out to evaluate cell proliferation, added into each well and the culture plates were incubated at 37°C with 5% CO_2_ for 1 h. The absorbance was detected using a microplate reader (Bio-Rad Laboratories, Richmond, CA, USA) at 450 nm

### 2.5 Transwell invasion test

The migratory and invasiveness were assessed using an 8-µm pore polycarbonate membrane Boyden chamber insert in a Corning Transwell apparatus (Corning, NY, USA). KLE and HEC-1B cells (5 × 104 cells) were plated into the upper compartment of chamber insets and lower compartments were filled with 500 µL DMEM containing 10% FBS. Cells were collected at 48 h post-transfection, washed with PBS and mechanically dissociated into a single-cell suspension. After 48 h of incubation, cells were fixed with 100% methanol, stained with 0.05% crystal violet, washed with PBS, invasion was observed under an inverted light microscope.

### 2.6 Luciferase reporter assay

Using Lipofectamine 2000, cells were transfected with miR-195-5p, circWEE1 3`-UTR-wild type, and mutant plasmids (Biomics Biotechnologies Co., Ltd. Nantong, China). Next, cells were transfected with miR-195-5p, VEGF 3`-UTR-wild type, and mutant plasmids (Biomics Biotechnologies Co., Ltd. Nantong, China) Lipofectamine 2000. Cells were incubated at 37°C 5% CO2 condition and transfected for 48 h. Renilla luciferase activity was acted as the control. The activity was detected by using a luciferase assay kit (Beyotime Institute of Biotechnology, Shanghai, China). The *Renilla* luciferase activity was normalized to that of the firefly luciferase activity.

### 2.7 Western blot analysis assay

The protein concentration was determined using the BCA Protein Assay Kit(). Protein was separated with sodium dodecyl sulfate polyacrylamide gel electrophoresis, transferred to a polyvinylidene difluoride (PVDF) membrane. The membrane was blocked with 5% nonfat milk in TBST for 1 h and incubated with WEE1 (ab137377, 1:1000, Abcam), EIF4A3 (ab32485, 1:1000, Abcam), VEGF (sc-7269, 1:1000, Santa Cruz Biotechnology), PI3K (sc-293,172, 1:1000, Santa Cruz Biotechnology), p-Akt (4060, 1:1000, Cell Signaling Technology, Inc.), Akt (4685, 1:1000, Cell Signaling Technology, Inc.) and GAPDH monoclonal anti-body (ab32441, 1:2000, Abcam) at 4°C overnight. Membrane was washed with PBS and incubated with the mouse ant-rabbit secondary antibody (sc-2004, 1:5000, Santa Cruz Biotechnology) at 37°C for 1 h. The immune complexes were detected using the ECL Western blot analysis Kit (Pierce Chemical) and analzyed using Image Lab 3.0 (Bio-Rad Laboratories, Inc.).

### 2.8 Flow cytometry for apoptosis analysis

Cells (1 × 10^6^ cells/well) were seeded into a 96-well plate at 37°C and Cells were washed with PBS. Cells were incubated at room temperature in the dark for 15 min, 5 mL Annexin V-FITC, and 5 mL PI. The apoptotic cells were measured using the FACScan flow cytometer (Becton, CA) equipped with CellQuest Software (Becton Dickinson).

### 2.9 Immunoprecipitation

RNA binding protein immunoprecipitation (RIP) assay was performed using an EZMagna RIP kit (Millipore, Billerica, MA, USA). 500 μg of total cellular protein were incubated with RIP buffer and were incubated with Proteinase K and magnetic beads conjugated with anti-eIF4A3 antibody or control (IgG). The immune-complex was exposed to western blotting.

### 2.10 In vivo *model*

Five-week-old BALB/c male nude mice (n = 12/every group) were provided by the laboratory animal facility of Yangzhou Medical University. The mice were reared at a temperature 22 ± 2°C and relative humidity 50 ± 5%, with 12-h light and 12-h dark alternation and allowed free access to food and water. BALB/c nude mice were intraperitoneally injected with pentobarbital sodium (40 mg/kg) and inoculated subcutaneously from the right forelimb with 0.2 mL of KLE (2 × 106 cells/mL) as reference. Every three days, tumor volume was measured using vernier caliper. All methods were carried out in accordance with relevant guidelines and regulations. All protocol for animals were approved by ethics committee of Yijishan Hospital of Wannan Medical College.

### 2.11 Immunofluorescence

Cell samples were fixed in 4% paraformaldehyde, incubated with 0.25% Tris-X100 for 10 min at room temperature for permeabilization. Cell samples were blocked with 5% BSA in PBST for 1 h at room temperature and incubated with anti- WEE1 or anti-EIF4A3 antibody (1:100, Abcam, UK), at 4°C overnight. After washing with TBST for three times, sections were incubated with secondary peroxidase-conjugated goat anti-rabbit-555 IgG (1:100, Santa Cruz Biotechnology) or goat anti-mouse-488 IgG (1:100, Santa Cruz Biotechnology) antibody for 2 h at room temperature. After washing with PBST for three times, sections were stained with DAPI for 15 min at darkness. Cell samples were observed using fluorescence microscope (Zeiss Axio Observer A1, Germany).

### 2.12 Immunohistochemical staining

The tumor tissue samples were fixed with 4% paraformaldehyde for 24 h and embedded in paraffin. For the immunohistochemical examination, the tissue sections (5 μm) were incubated with the VEGF (1:100) and WEE1 (1:100) antibodies. Tissue samples were observed using fluorescence microscope (Zeiss Axio Observer A1, Germany).

### 2.13 RNA-FISH

The cells were fixed with 4% paraformaldehyde at room temperature. The cells were incubated with 70% ethanol for 1 h at 4°C. Next, the stock solution of RNA probes was incubated with hybridization buffer (Ambion, Austin, TX, USA) overnight at 37°C, according to the manufacturer’s instructions for the RNA-FISH kit (RiboBio). After completing these steps, the nuclei were stained with DAPI (Invitrogen, Waltham, MA, USA). The cells were visualized and photographed using a laser confocal microscope (Olympus, Tokyo, Japan) after adding the fluorescence-quenching agent.

### 2.14 Statistical analyses

All data are presented as mean ± standard deviation. Shapiro Wilk test was performed to check the normal distribution of the data. Statistical differences were analyzed using Student’s t-test or one-way analysis of variance (ANOVA) and Tukey’s post test. Significance level was set as p < 0.05.

## 3. Results

The expression of circWEE1 and EIF4A3 levels were increased in patients with EC. Over-expression of circWEE1 or down-regulation of miR-195-5p promoted cell migration and proliferation in EC. Next, we verified that eIF4A3 binds to the circWEE1 mRNA transcript, circWEE1 served as a sponge that directly targeted miR-195-5p. Bioinformatics prediction forecast that miR-195-5p directly targeted VEGF at 3’-UTR, which was confirmed by luciferase reporter assay.

### 3.1 Up-regulation of circular RNA hsa circWEE1 indicates cell proliferation, migration, and invasion in EC

To analyze the changes of Circular RNA in patients with EC, we used PCR to measure the expression of Circular RNA in patients with EC. As shown in Figure 1a, circWEE1 expression levels was increased in patients with EC, compared with negative group. CircWEE1 expression levels in normal group was lower than those of in patients with I–II EC, circWEE1 expression levels in patients with I–II EC, was lower than those of in patients with III EC, circWEE1 expression levels in patients with III EC, was lower than those of in patients with IV EC (p < 0.05) (Figure 1b). CircWEE1 expression in KLE cells were increased, compared with NHA (Figure 1c). The study explained the effects of circWEE1 on cell proliferation, migration, and invasion in EC. CircWEE mimics increased circWEE expression and promoted cell proliferation in KLE cell, compared with negative group (p < 0.05) (Figure 1d-e). CircWEE inhibitor mimics decreased circWEE expression and reduced cell proliferation in HEC-1B cell, compared with negative group (figure 1f-g). Over-expression of circWEE promoted cell migration and reduced apoptosis in KLE cell, compared with negative group (Figure 1h-k). However, down-regulation of circWEE reduced cell migration and induced apoptosis in HEC-1B cell, compared with negative group (p < 0.05) (Figure 1l-o), suggesting that circWEE1 take part in cell migration and proliferation in EC.

**Figure 1.** Circular RNA has circWEE1 in patients with EC and indicates cell proliferation, migration and invasion in EC. CircWEE1 expression levels in patients with EC (A), circWEE1 expression in clinical stages of patients with EC (B), circWEE1 expression (C) in EC cell lines than in the cell line (NHA), CircWEE1 increased the expression levels of circWEE1 (D) and cell proliferation (E), circWEE1 inhibitor the expression levels of circWEE1 (F) and cell proliferation (G), over-expression of circWEE1 promoted migration (H and I) and inhibited apoptosis (J and K); down-regulation of circWEE1 reduced migration (L and M) and increased apoptosis (N and O). The transfection effects were confirmed by using qRT-PCR method. Negative, negative mimics group; WEE1 inhibitor, down-regulation of circWEE1 expression group; WEE1, over-expression of circWEE1 expression group. **p < 0.01 versus normal group or NHA group or **p < 0.01 versus negative mimics group.

*Circular RNA hsa circWEE1 regulates miR-195-5p*

To analyze the mechanism of circWEE1 on cell proliferation, migration, and invasion in EC, we used gene chip to analyze the circWEE1 regulates the changes of microRNA *in vitro* model. MiR-195-5p expression may be target spot for circWEE1 (Figure 2a-b). As shown in Figure 2c, there was a negative correlation between circWEE1 and miR-195-5p. The putative-binding sites of miR-195-5p on the circWEE1 wild-type (WT) or mutated sequence are shown and luciferase reporter activity was reduced in miR-195-5p+ circWEE1-WT, compared with negative group (p < 0.05) (Figure 2d-f). Subcellular analysis demonstrated the circWEE1 in the cytoplasm or nuclear material in KLE cells (Figure 2g). RNA-FISH demonstrated the distribution of circWEE1 and miR-195-5p in cytoplasm and nuclear material (Figure h). MiR-195-5p expression may be target spot for circWEE1.

**Figure 2.** Circular RNA hsa circWEE1 regulates miR-195-5p. Heat map (A) and analyze map (B) of microarray analysis, there was a negative correlation between circWEE1 and miR-195-5p (C), 3’-UTR of circWEE1 is complementary to the miR-195-5p seed sequence (D), luciferase reporter activity (E and F), Subcellular analysis demonstrated the circWEE1 in the cytoplasm or nuclear material in KLE cells (G), RNA-FISH demonstrated the distribution of circWEE1 and miR-195-5p in cytoplasm and nuclear material (H). Negative, negative mimics group; miR-195-5p+circWEE1-wt, circWEE1 expression and circWEE1-wt group; miR-195-5p+circWEE1-mut, circWEE1 expression and circWEE1-mut group. **p < 0.01 versus negative mimics group.

### 3.2 CircWEE1 accelerates cell proliferation and migration by targeting miR-195-5p

The study explained the mechanism of circWEE1 on cell proliferation and migration of EC. We found that miR-195-5p mimics increased the expression of miR-195-5p, and reduced cell proliferation in KLE cell, compared with negative group (Figure 3a-b). Si-miR-195-5p mimics decreased the expression of miR-195-5p, and promoted cell proliferation in KLE cell, compared with negative group (p < 0.05) (Figure 3c-d). Over-expression of miR-195-5p reduced cell migration, and down-regulation of miR-195-5p promoted cell migration, compared with negative group (Figure 3e-h). Then, over-expression of miR-195-5p increased apoptosis, and down-regulation of miR-195-5p reduced apoptosis, compared with negative group (p < 0.05) (Figure 3i-l). The induction of miR-195-5p suppressed VEGFA, PI3K, and p-Akt protein expressions in KLE cells following over-expression of circWEE1, compared with over-expression of circWEE1 (Figure 3m). The induction of miR-195-5p reduced cell proliferation and cell migration, and increased apoptosis in KLE cells following over-expression of circWEE1, compared with over-expression of circWEE1 (p < 0.05) (Figure 3n-3r). These results suggest that circWEE1 accelerates cell proliferation and migration by targeting miR-195-5p.

**Figure 3.** CircWEE1 accelerates cell proliferation and migration by targeting miR-195-5p. CircWEE1 increased the expression levels of circWEE1 (A) and cell proliferation (B), circWEE1 inhibitor the expression levels of circWEE1 (C) and cell proliferation (D), over-expression of circWEE1 promoted migration (E and F) and inhibited apoptosis (G and H); down-regulation of circWEE1 reduced migration (I and J) and increased apoptosis (K and L), VEGF, PI3K, p-Akt and Akt protein expression (M), cell proliferation (N), migration (O and P), apoptosis (Q and R). Negative, negative mimics group; circWEE1, over-expression of circWEE1 expression group; circWEE1+ micR-195-5p, over-expression of circWEE1 expression and micR-195-5p group. **p < 0.01 versus negative mimics group, ^##^p < 0.01 versus over-expression of circWEE1 group.

### 3.3 CircWEE1 promotes eIF4A3 expression

The data from an RIP (RNA binding protein immunoprecipitation) assay using anti-eIF4A3 antibody indicated that circWEE1 can bind with eIF4A3 mRNA (Figure 4a). Up-regulation of eIF4A3-induced WEE1 mRNA expression, and down-regulation of eIF4A3 reduced WEE1 mRNA expression in KLE and HEC-1B cells, compared with negative group (p < 0.05) (Figure 4b-c). The results of immunofluorescence showed that eIF4A3 promoted eIF4A3 and WEE1 expression *in vitro* model, compared with negative group (p < 0.05) (Figure 4d). Si-eIF4A3 suppressed eIF4A3, VEGFA, PI3K, and p-Akt protein expressions in KLE cells following over-expression of circWEE1, compared with over-expression of circWEE1 (Figure 4e). The inhibition of eIF4A3 reduced cell proliferation and cell migration, and promoted apoptosis in KLE cells following over-expression of circWEE1, compared with over-expression of circWEE1 (figure 4f-j).

**Figure 4.** CircWEE1 promotes eIF4A3 expression. RIP (A), WEE1 mRNA expression (B and C), Immunofluorescence (D), VEGF, PI3K, p-Akt, and Akt protein expression (E), cell proliferation (F), migration (G and H), apoptosis (I and J). Negative, negative mimics group; circWEE1, over-expression of circWEE1 expression group; circWEE1+ micR-195-5p, over-expression of circWEE1 expression and micR-195-5p group. **p < 0.01 versus negative mimics group, ^##^p < 0.01 versus over-expression of circWEE1 group.

### 3.4 CircWEE1 up-regulates VEGFA expression via miR-195-5p

This study used bioinformatics method (http://www.targetscan.org) to explain binding sites. As shown in Figure 5a, the putative-binding sites of miR-195-5p on the VEGFA wild-type (WT) or mutated sequence are shown and luciferase reporter activity was reduced in miR-195-5p + VEGFA-WT, compared with negative group (Figure 5a-c). Then, over-expression of miR-195-5p-induced VEGFA, PI3K, and p-Akt protein expressions in HEC-1B cells, compared with negative group (Figure 5d). Si-miR-195-5p suppressed VEGFA, PI3K, and p-Akt protein expressions in KLE cells, compared with negative group (Figure 5e). Next, si- VEGF suppressed VEGFA, PI3K, and p-Akt protein expressions in HEC-1B cells following over-expression of circWEE1, compared with over-expression of circWEE1 (p < 0.05) (figure 5f). The inhibition of VEGF reduced cell proliferation and cell migration, and promoted apoptosis in KLE cells following over-expression of circWEE1, compared with over-expression of circWEE1 (Figure 5g-k). These results show that VEGFA is participated into the effects of CircWEE1 on EC growth by EC growth.

**Figure 5.** CircWEE1 up-regulates VEGFA expression via miR-195-5p. 3’-UTR of VEGFA is complementary to the miR-195-5p seed sequence (A), luciferase activity levels (B and C), VEGF, PI3K, p-Akt, and Akt protein expression (D, E, and F), cell proliferation (G), migration (H and I), apoptosis (J and K). Negative, negative mimics group; circWEE1, over-expression of circWEE1 expression group; circWEE1+ si-EIF4A3, over-expression of circWEE1 expression and si-EIF4A3 group. **p < 0.01 versus negative mimics group, ^##^p < 0.01 versus over-expression of circWEE1 group.

### 3.5 *CircWEE1 enhances EC growth* in vivo *by miR-195-5p*

In vivo, U87 cells were transfected with the mock or circWEE1 plasmid or si- miR-195-5p. The results indicated that the overexpression of circWEE1 generated an outstanding increase tumor volume, tumor size, and tumor weight *in vivo* model (Figure 6a-6d). IHC assay data showed that over-expression of circWEE1 promoted EIF4A3 protein expression *in vivo* model (Figure 6e). We found that over-expression of circWEE1-induced circWEE1, EIF4A3, VEGF, PI3K, and p-Akt protein expression *in vivo* model (figure 6f). Next, si- miR-195-5p also promoted tumor growth, tumor volume, tumor size, and tumor weight *in vivo* model (Figure 6g-j). IHC assay data showed that Silencing -miR-195-5p-induced VEGF protein expression *in vivo* model (Figure 6k). Silencing-miR-195-5p induced VEGF, PI3K, and p-Akt protein expression *in vivo* model (Figure 6l), suggesting that CircWEE1 may enhance EC growth.

**Figure 6.** CircWEE1 enhances EC growth in vivo by miR-195-5p. Tumor volume (A and B), Tumor size (C), Tumor weight (D), WEE1 expression (E), WEE1, EIF4A3, VEGF, PI3K, p-Akt, and Akt protein expression (D, E, and F) by circWEE1; Tumor volume (G and H), Tumor size (I), Tumor weight (J), WEE1 expression (K), WEE1, EIF4A3, VEGF, PI3K, p-Akt, and Akt protein expression (L) by si-miR-195-5p. Negative, negative mimics group; circWEE1, over-expression of circWEE1 expression group; si-miR-195-5p, down-regulation of miR-195-5p expression group. **p < 0.01 versus negative mimics group.

## 4. Discussion

EC in the United States, Europe, and other developed areas, is close to 50% of new gynecological malignancies [20]. In 2018, there were 54,870 new cases of EC in the United States, and 10,170 deaths In recent years, with the rapid economic development, people’s habits and diet structure has changed greatly [21]. With the increase of metabolic diseases, EC also has a trend of increasing incidence rate and younger onset [22]. According to the etiology and epidemiological data of EC, the high-risk factors of EC can be roughly divided into four categories: one is related to genetic materials; the other is anatomical and physiological conditions are basically normal; the third is obvious disease state, namely the effect of endogenous estrogen; the fourth is external factors [23–25]. In our study, we found that circWEE1 (circWEE1) expression levels were increased in patients with EC. Up-regulation of circular RNA hsa circWEE1 indicates cell proliferation, migration, and invasion in EC. Yuan et al. showed that inhibition of WEE1 suppresses the tumor growth in laryngeal squamous cell carcinoma [26]. These data highlight a novel oncogenic function of circRNA in EC tumorigenesis. In future studies, we need to assess more EC tissues to confirm the oncogenic role of circWEE1.

A large number of studies have shown that the expression levels of various miRNAs are abnormally changed in EC tissues or cells [27]. Some miRNAs act as oncogenes, while others act as tumor suppressor genes, playing an important role in the occurrence and progression of EC [27]. These miRNAs are expected to be novel markers for the diagnosis and prognosis of EC, and also provide new ideas and targets for the development of anti-tumor drugs [28]. However, there are complicated network interactions between miRNAs and transcriptional factors that regulate their transcription, their target mRs, and miRs [28]. Thus, further studies are necessary to elucidate the role and mechanism of miRs in EC. At present, circWEE1 accelerates cell proliferation and migration of EC by targeting miR-195-5p. Lin et al. reported that miR-195-5p suppressed GATA3-mediated IL-4 secretion in colorectal cancer cells [29]. Those analysis results suggest that circWEE1 may play roles in EC by interacting with miR-195-5p.

The binding of VEGF to VEGFR-2 would promote VEGF-mediated endothelial cell proliferation, promote endothelial cell survival and anti-apoptosis, promote endothelial cell migration, and increase vascular permeability [30]. These functions have been dominant in the field of VEGF research since the clearly established role of VEGF in promoting angiogenesis and lymphangiogenesis [31]. In addition, these studies have profound insights and understanding of the complex processes and mechanisms of angiogenesis [31]. Importantly, these studies are considered as the foundation for the development of targeted therapies for VEGF and VEGFR [30]. In this study, we demonstrated that circWEE1 up-regulates VEGFA expression via miR-195-5p. Sandrim et al. concluded that miR-195-5p may contribute to decreased expression of VEGFA in endothelial cell cultures incubated with preeclampsia plasma [32]. Thus, miR-195-5p/VEGFA could observably impact the EC phenotype.

Based on the ‘sponge’ effect of circRNA molecules on miRNA, their expression is associated with the occurrence and progression of various diseases, and significantly different expression can be observed in pathological samples [27]. Studies have shown that miR-7 plays an important role in nervous system diseases, diabetes, and various cancers [16,33]. Therefore, the relationship between circRNA and these diseases is also of great significance. Among them, some studies have confirmed that Cdr1as affects the occurrence and progression of relevant diseases by regulating the expression of miR-7 [33]. In addition to miR-7, circRNA has also been found to interact with other miRNAs in disease [34]. Moreover, multiple studies have also found that the expression of circRNA is significantly different in disease [34,35]. In the present study, we found a novel circRNA, circWEE1, that may serve as an oncogene in EC. Wu et al. indicated that miR-526b-3p may target WEE1and inhibit EC tumorigenesis and progression [36]. Therefore, it might be explained that circWEE1 exerts physiological functions through sponging miR-195-5p/VEGFA.

Studying the different functions of eIF4A1, eIF4A2 and eIF4A3 is a focus of recent eIF4A research [8]. In consideration of their 90% similarity, it is critical to elucidate the molecular mechanisms by which these two proteins are recruited to different protein complexes [37]. Abnormal protein synthesis caused by uncontrolled expression of the translation initiation complex factor eIF4F is a common cause of malignant tumors in humans [38]. eIF4A is the most abundant subunit of eIF4F with RNA-dependent ATPase and RNA helicase activity, playing an important role in the initiation of protein synthesis [39] Studies have demonstrated that eIF4A3 is overexpressed in a variety of tumors, including melanoma, hepatocellular carcinoma, and lymphoma [38,39]. In this study, we found that circWEE1 promotes eIF4A3 expression, and the inhibition of eIF4A3 reduced the effects of circWEE1 on cell proliferation and migration of EC. Therefore, we concluded that eIF4A3 can induce circWEE1 cyclic formation. The mechanism between CircWEE1, EIF4A3 and miR-195-5 was not clear, we will further research it.

## 5. Conclusion

We first identified that circWEE1 acts as an oncogene and promotes EC cell proliferation and migration. EIF4A3-induced circWEE1 cyclization and increased circWEE1 expression. CircWEE1 can directly bind to miR-195-5p and regulate its expression. We demonstrated that VEGF is target genes of the circWEE1/miR-195-5p axis in EC cells (Figure 7). Furthermore, our results indicated that a solid basis to develop a better understanding of EC pathology and identify potential therapeutic targets for the treatment of EC.

**Figure 7.** Circular RNA hsa circ (circWEE1)/ EIF4A3 promoted cell migration and proliferation in EC via VEGF signaling by miR-195-5p.

## Data Availability

The datasets used or analysed during the current study are available from the corresponding author on reasonable request.
